# An Intelligent Heartbeat Classification System Based on Attributable Features with AdaBoost+Random Forest Algorithm

**DOI:** 10.1155/2021/9913127

**Published:** 2021-07-09

**Authors:** Runchuan Li, Wenzhi Zhang, Shengya Shen, Jinliang Yao, Bicao Li, Bing Zhou, Gang Chen, Zongmin Wang

**Affiliations:** ^1^School of Information Engineering, Zhengzhou University, Zhengzhou 450000, China; ^2^Cooperative Innovation Center for Internet Healthcare, Zhengzhou University, Zhengzhou 450000, China; ^3^Foreign Languages Department, Zhengzhou University of Economics and Business, Zhengzhou, Henan 450000, China; ^4^Electric and Information Engineering, Zhongyuan University of Technology, Zhengzhou, Henan 450000, China

## Abstract

Arrhythmia is a common cardiovascular disease that can threaten human life. In order to assist doctors in accurately diagnosing arrhythmia, an intelligent heartbeat classification system based on the selected optimal feature sets and AdaBoost + Random Forest model is developed. This system can acquire ECG signals through the Holter and transmit them to the cloud platform for preprocessing and feature extraction, and the features are input into AdaBoost + Random Forest for heartbeat classification. The analysis results are output in the form of reports. In this system, by comparing and analyzing the classification accuracy of different feature sets and classifiers, the optimal classification algorithm is obtained and applied to the system. The algorithm accuracy of the system is tested based on the MIT-BIH data set. The result shows that AdaBoost + Random Forest achieved 99.11% accuracy with optimal feature sets. The intelligent heartbeat classification system based on this algorithm has also achieved good results on clinical data.

## 1. Introduction

In recent years, the incidence rate of cardiovascular diseases is increasing, which seriously threatens human life [1]. Arrhythmia can be divided into two types, life-threatening arrhythmia and nonlife-threatening arrhythmia. Life-threatening arrhythmia can lead to cardiac arrest and sudden death. These patients need urgent treatment. Although nonlife-threatening arrhythmia may not threaten human life immediately, it still needs to be treated timely to avoid further deterioration. Therefore, the intelligent detection and diagnosis of arrhythmia is of great significance for monitoring, preventing the occurrence of heart disease, and improving the work efficiency of doctors.

Long-term continuous monitoring [2, 3] of electrocardiogram (ECG) provides valuable information for the prevention of heart attack diseases [4]. Doctors can diagnose the nature of arrhythmia by analyzing the ECG. In order to monitor the nature of abnormal heartbeat, it is necessary to analyze the electrical signal of each heartbeat. However, analyzing long-term ECG records is very time-consuming for doctors. Sometimes, doctors may inevitably make personal mistakes. Therefore, accurate intelligent classification of arrhythmia can improve doctors' efficiency and reduce the occurrence of misdiagnosis or missed diagnosis [5].

This paper presents a heartbeat classification system based on multiple-feature fusion and improved random forest, which can classify arrhythmia from real data collected by the ECG acquisition equipment. This system completely accomplished the process from ECG signal collection to heartbeat classification, and then to present the classification results to doctor. The contribution of this research presented in this paper is as follows:

1. Developed an intelligent heartbeat classification system from collection, analysis, to result presentation. This system can effectively improve doctors' work efficiency.
2. An optimal attributable heartbeat feature set is obtained towards the best possible heartbeat classification system via feature comparison identified through the implementation of multiple classifiers, arrhythmia classification analysis, and feature combination comparison.
3. After testing, AdaBoost + Random Forest was found to be the best heartbeat classification system. This method can not only deal with input samples with high-dimensional characteristics but also effectively deal with imbalance data classification with random forest approach, which provided an effective method to balance the error of the data set.
4. The interpretability analysis of the learning content of heartbeat classification system based on AdaBoost + Random Forest algorithm is carried out by constructing feature sets of different ECG prior knowledge and improving the accuracy of heartbeat classification, which has important clinical significance.

The rest of this paper is organized as follows: Part 2 briefly introduces the related work. Part 3 provides an over-view of the system architecture. Part 4 details the major process of our system, the algorithm of heartbeat classification. Part 5 presents system performance analysis. Part 6 summarizes the full text.

## 2. Related Work

In the past, the diagnosis of arrhythmia was mainly dependent on the experience of doctors. With the development of artificial intelligence, automatic classification has been applied to various industries in recent years [6–9]. A variety of systems for automatic classification of heartbeat had been proposed by some researchers. These systems can be divided into two types, a classification system based on deep learning and a classification system based on feature engineering.

A few systems [10–14] used deep neural network to classify heartbeat, but deep neural networks (DNN) have problems with parameter redundancy. Hilera et al. [15] used ANN to detect arrhythmia to study the usefulness of ANN in clinical diagnosis. But, it is difficult to accurately analyze the performance indicators of neural network using ANN. Li et al. [16] merged the shape and rhythm of the heartbeat into a two-dimensional information vector, and used Convolutional Neural Network to classify the heartbeat. The results show that the system has a better classification effect on *v* and *s* categories. Wang et al. [17] proposed a globally updatable classification system in view of the large individual differences and the high cost of marking the ECG icon, which has a good classification effect. The algorithm of heartbeat classification based on deep learning can effectively distinguish between different types of arrhythmias. It is very important for doctors to diagnose diseases, as precise analytical classification can help doctors to accurately diagnose and accurately draw up appropriate treatment plans. However, methods based on deep learning cannot analyze the impact of features on the performance of heartbeat classification.

Feature extraction is an important step in the accurate classification of arrhythmia. Over the past few decades, researchers have used a variety of features to automatically classify arrhythmia, including ECG morphology [18, 19], interval [20–23], QRS area [24, 25], wavelet coefficient [26, 27], hermite coefficient [28], and high-order statistics [28, 29]. The relevant features of ECG signals are extracted, and then input into learning algorithms to induce models to classify arrhythmia. At present, machine learning is widely used in medical diagnosis to assist doctors improve the efficiency of diagnosis and treatment. Yildirim [30] uses the wavelet transform method to detect heartbeats in ECG data, and divides these heartbeats into segments according to certain cycles, and then performs multi-resolution wavelet transforms into the segmented signals to obtain different frequencies of the wavelet coefficients, and then develop a heartbeat classification system. The test results confirm the effectiveness of this approach. However, this method only focuses on the features of wavelet coefficients and does not concentrate on other features, which provides a good potential for further improvement. Alickovic and Subasi [31] applied Random Forest to the diagnosis of ECG arrhythmia, using Discrete Wavelet Transform to decompose the ECG signal into different continuous frequency bands, and the purpose of ECG intelligent diagnosis system is to distinguish each kind of heartbeat accurately. The above work has made some achievements in heartbeat classification using morphological features, interval features, QRS wave area, wavelet coefficients, and other aspects, and these intuitive features make full use of the doctor's logical experience and ECG data. There is an expectation in improving heart rate classification accuracy.

The project depends on the combination of intuitive attributive features. In order to select the best feature combination, the influence of different feature combinations of heartbeat classification is analyzed. A new heartbeat classification system based on attributable intelligent classification method is presented in this paper. It improves the accuracy of classification and the work efficiency of doctors.

## 3. System Architecture

The fundamental purpose of the ECG intelligent diagnosis system is to distinguish each kind of heartbeat accurately. There is an expectation in improving heart rate classification accuracy. The research value of this project depends on the effective selection and combination of intuitive attributive features, as well as the interpretable reasoning analysis of classification performance. A new heartbeat classification system based on multi-feature fusion and AdaBoost + Random Forest method is presented in this paper. In order to select the best feature combination, the influence of different feature combinations on heartbeat classification is analyzed. The best feature combination is selected and input into AdaBoost + Random Forest for classification. It effectively uses the ECG data and improves the accuracy of classification. The focus of the system is heartbeat classification system based on attributable features and AdaBoost + Random Forest algorithm; the next section will describe the system process in detail. This section introduces the overall structure of the system.

The overall architecture of the system is shown in Figure 1. It shows that the system components mainly include Holter, smart phones, and soft system. The data collected through Holter is uploaded to the server for analysis. This process requires the user to download the APP on the mobile phone. Before classification, the system automatically extracts features based on denoised ECG data. These features are the best combination of features selected after the test. Compared with other systems, the classification system based on these features makes full and effective use of ECG data and has better interpretability. After classification, the result report will be sent to the patient after being checked by a doctor.  Figure 2 is the logical design of the system.

Figure 3 shows the ECG system function diagram. The system is developed based on Microservice [32], which has better scalability, easy deployment, and low coupling. The holter collects data from the patient and transmits the data to the subject's mobile phone via Bluetooth. The acquired data are stored in the ECG parameter center on the cloud platform through the http/https protocol, namely, ECGDatabaseGateway Server. The specific transmission, storage, and analysis steps of the collected ECG data on the cloud platform are as follows: ECGDeviceGateway receives and distributes ECG data; ECGDataRouter server realizes the forwarding of ECG data through the subscription-publishing mechanism through NATS. ECGAnalyzeGateway sends the ECG data analysis request to ECGAnalyzeServer that deploys the core algorithm proposed. After receiving the request, ECGAnalyzeServer passes the ECG parameters to the algorithm program for analysis. The transmission uses RPC [33] in order to achieve high transmission efficiency and low performance consumption. The ECGAnalyzeGateway server uses NATS [34] to transmit the analyzed results to the ECGPipeGateway server for real-time transmission during diagnosis. The ECGPipeGateway server displays the results of real-time ECG monitoring on each terminal through the WebSocket protocol [35] that can unilaterally send information to the client, reducing the delay caused by waiting for a reply. At the same time, ECGAnalyzeServer transmits the results to the ECGDataBaseGateway server, which is responsible for storing results of the ECG analysis and classification. Due to the complexity of ECG data, MongoDB [36] is used to store ECG data.

## 4. System Process

This process uses multi-feature fusion and AdaBoost + Random Forest method to classify heartbeats. It includes ECG signal data, preprocessing, feature extraction, and heartbeat classification.  Figure 4 shows the framework of heartbeat classification algorithm.

### 4.1. ECG Signal Preprocessing

In order to classify heartbeat more accurately, it is necessary to denoise the ECG data and detect waveform. The wavelet transform can retain the features and important physiological details of ECG signal, and have a simple calculation process [37]. Therefore, a continuous wavelet is used to remove the original ECG signal noise and detect the boundaries and peak positions of the three waves. In this paper, wavelet transform is a signal time-frequency analysis method [38], which provides time-domain and frequency-domain features. The principle of continuous wavelet transform [39] is shown in formulas (1) and (2). (1) and (2). This paper uses wavelet transform to achieve denoising and R wave detection.

(1) $$\begin{array}{c} W_{f}\left(a,\tau \right)=a^{-1/2}\int_{-\infty }^{+\infty }f\left(t\right)\psi \left(\frac{t-b}{a}\right)\text{d}t, \end{array}$$

(2) $$\begin{array}{c} \psi_{a,\tau }\left(t\right)=a^{-\left(1/2\right)}\psi \left(\frac{t-b}{a}\right),\;a>0,\tau \in R. \end{array}$$

In formula (1), *a* is the scale factor, and *b* is the transform factor. Their role is to stretch the basic wavelet function *ψ*(*t*); *τ* reflects the displacement, and *a* and *τ* are continuous variables. The results of CWT can be expressed as functions of scale factor *a* and transformation factor *b*. The translation factor enables the wavelet to complete the ergodic analysis along the time axis of the signal. The transform factor can approach different frequency signals in every traversal through scaling wavelet transform.

### 4.2. Heartbeat Feature Extraction and Combination

A complete cardiogram consists of P wave, QRS wave, and T wave. The time interval between the feature points of these waves directly reflects the systolic and diastolic process of heart atrium and ventricle, which is of great value in the diagnosis of heart disease [40]. The extracted ECG features are described as follows:

In this paper, the sampling rate is 360 Hz. According to the R peak position, 235 single heartbeat morphological features are extracted [41]. Among them, there are 90 sampling points before the R peak and 144 sampling points after the R peak. If there are less than 235 sampling points before and after the first or last QRS complex is detected in the ECG record file, the corresponding heartbeat is ignored. Each record in the MIT-BIH arrhythmia database contains two leads, of which lead A is lead II and lead B is lead V1. However, in some records, lead B is known to be V2, V5, or V4. According to literature [41, 42], QRS complex is more prominent in lead A, so lead A is usually used to detect heartbeat, lead B has more advantages in distinguishing S and V category arrhythmia. A total of 470 single heartbeat morphological features are obtained from two leads, respectively.  Figure 5 shows the two leads in an MIT-BIH arrhythmia database record 210 (10 sec).

P wave interval, QRS wave interval, T wave interval, PR segment, ST-T interval, QT interval, and RR interval are common features of ECG. The sampling rate (SR) is 360 Hz in this study.  Figure 6 is the interval diagram of normal heartbeat. The calculation formula is shown in equations (3)– (9):

(3) $$\begin{array}{c} P\text{ wave interval}=\frac{P_{\text{end}}\;-P_{\text{start}}}{\text{SR}}, \end{array}$$

(4) $$\begin{array}{c} \text{QRS wave interval}=\frac{{\text{QRS}}_{\text{end}}\;-{\text{QRS}}_{\text{start}}}{\text{SR}}, \end{array}$$

(5) $$\begin{array}{c} T\text{ wave interval}=\frac{T_{\text{end}}\;-T_{\text{start}}}{\text{SR }}, \end{array}$$

(6) $$\begin{array}{c} \text{PR segment}=\frac{{\text{QRS}}_{\text{start}}\;-P_{\text{end}}}{\text{SR}}, \end{array}$$

(7) $$\begin{array}{c} \text{ST}-T\text{ intervel}=\frac{T_{\text{end}}\;-{\text{QRS}}_{\text{end}}}{\text{SR}}, \end{array}$$

(8) $$\begin{array}{c} \text{QT interval}=\frac{T_{\text{end}}\;-{\text{QRS}}_{\text{start}}}{\text{SR}}, \end{array}$$

(9) $$\begin{array}{c} \text{RR interval}=\frac{R_{\text{next peak}}\;-R_{\text{current peak}}}{\text{SR}}. \end{array}$$

The QRS complex is the most energetic part of the ECG signal and contains most of the information of the entire heartbeat. The time from the start of the QRS complex to the end of the QRS complex is the QRS time limit, and the QRS wave area is the integral sum of the QRS complex from the start to the end.

The QRS complex reflects the changes in left and right ventricular depolarization potentials and time. The first downward wave is the Q wave, the upward wave is the R wave, and the downward wave is the S wave. Therefore, the shape of the QRS complex is mainly considered when selecting the wavelet base. According to the waveform of a cardiac cycle, we choose the db6 wavelet as the wavelet basis function to implement wavelet decomposition [43], because the db6 wavelet has good regularity, which makes the reconstructed signal smooth. The frequency band of QRS complex is generally in the range of 0.5–45 Hz. The wavelet packet decomposition diagram is shown in Figures 7 and 8.  Figure 7 shows ECG original signal and its wavelet transform on a 1–6 scale.  Figure 8 shows ECG original signal and its wavelet transform on a 7–12 scale. S represents the input ECG signal, A represents the approximation coefficient of the wavelet packet decomposition, and D represents the detail coefficient of the wavelet packet decomposition. In this paper, the wavelet coefficients are extracted as features.

In feature engineering, as a single feature cannot fully describe the properties of ECG comprehensively, first-order discrete features are often combined to form high-order combined features, so as to improve the fitting ability of complex relationships. Therefore, the features are divided into five sets, namely, A, B, C, D, and E. Among them, set A and B are morphological features, set C is interval information, set D is area information, and set E is frequency feature. The definition and division of five feature sets are as follows:

  Set A: {235 single heartbeat morphological features from single lead}
  Set B: {470 single heartbeat morphological features from double leads}
  Set C: {P wave interval, QRS wave interval, T wave interval, PR segment, ST-T interval, QT interval, and RR interval}
  Set D: {QRS area}
  Set E: {Wavelet coefficient}

### 4.3. AdaBoost + Random Forest Model

AdaBoost ensemble algorithm is an iterative algorithm based on multiple base learners of the same type. The goal of iterative is to form a strong learner [44–46]. The algorithm trains different basic learners on the same training set, changes the weights of samples of iteration, and uses a weighted voting mechanism to stack multiple basic learners, and finally gets the best, strong learner for the overall classification performance.

The basic learner of AdaBoost + RF algorithm consists of random forest. Random forest is an important integrated learning method based on bagging. The final prediction result is based on a voting algorithm. Compared with other classification algorithms, random forest algorithm can maintain high accuracy and has good stability [47]. The steps in AdaBoost algorithm are described in Algorithm 1.  Figure 9 shows the process of generating the final classifier. Equations (10)–(13) refer to literature [45].

In AdaBoost ensemble algorithm, the training data set is *X*={(*x*_1_,  *y*_1_), (*x*_2_,  *y*_2_),…, (*x*_*N*_,  *y*_*N*_)}, where *x*_*i*_ represents the sample point and *y*_*i*_ represents the corresponding category of the sample; the importance of the basic classifier *G*_*m*_ depends on its error rate. The error rate *e*_*m*_ is defined as

(10) $$\begin{array}{c} e_{m}=\sum_{j=1}^{N}w_{j}I\left(C_{i}\left(x_{j}\right)\neq y_{j}\right), \end{array}$$

where {(*x*_*j*_, *y*_*j*_)*|j*=1,2,…, *N*} represents a set of N training samples. If the predicate P is true, then *I*(*p*)=1, otherwise 0. The base classifier is defined as

(11) $$\begin{array}{c} \alpha_{m}=\frac{1}{2}\ln\left(\frac{1-e_{m}}{e_{m}}\right). \end{array}$$

According to the definition of *α*_*m*_ and *e*_*m*_, the lower error rate means that the base classifier is more important. Once the *e*_*m*_ of a base classifier is higher than 50%, the weight of this round needs to be restored to the initial value and resampled. Update the weight distribution of the training data set:

(12) $$\begin{array}{c} w_{m+1,i}=\frac{w_{m,i}}{z_{m}}\exp\left(-\alpha_{m}y_{i}G_{m}\left(x_{i}\right)\right),\;i=1,2,\ldots ,N, \end{array}$$

where *z*_*m*_=∑_*i*=1_^*N*^*w*_*m*,*i*_exp(−*α*_*m*_*y*_*i*_*G*_*m*_(*x*_*i*_)) is the gauge factor that makes the sum of all *w* equal to 1. The final output function is

(13) $$\begin{array}{c} G\left(x\right)=\text{sign}\left(\sum_{m=1}^{M}\alpha_{m}G_{m}\left(x\right)\right). \end{array}$$

## 5. System Performance Assessment Analysis

The system test is implemented on Python 3.7 and MATLAB @ R2018b. Gaussian Naive Bayes (GNB), Linear Discriminant Analysis (LDA), Decision Tree (DT), Random Forest model (RF), Gradient Lifting Iterative Decision Tree (GBDT), Support Vector Machine (SVM), and Logistic Regression (LR) are selected for performance comparison. When the data are unbalanced, for the multi-classification problem, the type with a large sample size will have an over-fitting phenomenon during training, and the type with a small sample size will have an under-fitting phenomenon, resulting in false high accuracy of the overall heartbeat classification. This paper deals with data imbalance based on the algorithmic perspective and alleviates the problem of data imbalance by combining AdaBoost and Random Forest. Random Forests are relatively robust to missing data and unbalanced data, and can well predict the effects of up to thousands of variables [48]. The principle is to use small sample sizes in all classifications when generating the training set, and at the same time randomly extract data from the large sample size in the classification to combine with the small sample size to form the training set to obtain multiple training sets and decision tree models. Data imbalance can be effectively alleviated by integrating multiple decision trees. Adaboost can independently and randomly extract several subsets from the majority class, combine each subset with the minority class data to train to generate multiple base classifiers, and then weight them to form a new classifier. In this paper, comparing the performance of multiple classifiers, while considering the characteristics of the classifiers, a random forest is selected as the base classifier. Then, ensemble learning is used to alleviate data imbalance and improve classifier performance. This section mainly describes the test data, evaluation criteria, and presents 16 different test results tested on different sets of data with varied composition of heartbeat features. The results of different test are compared and analyzed. Clinical data are used to verify system performance.

### 5.1. Test Data

In this paper, all the tests are carried out on MIT-BIH arrhythmia database. The MIT-BIH arrhythmia database is a standard database to evaluate arrhythmia detection, and is widely used for algorithm verification. The database contains 48 records from 47 subjects. Each record contains two 30-minute ECG lead signals (lead A and lead B). In 48 records, 23 records included normal sinus rhythm (NSR) and a representative group of conventional arrhythmias; the other 25 records included uncommon but clinically significant cardiac abnormalities [49].

According to the ANSI/AAMI EC57 standard proposed by the Association for the advancement of medical instruments (AAMI), there are five categories proposed by AAMI in 2012-specific classification: N (nonectopic beats), S (supraventricular ectopic beats), V (ventricular ectopic beats), F (fusion beats), and Q (unknown beats) [50]. In this paper, 90% data of MIT-BIH arrhythmia database are randomly used for training set and 10% data of MIT-BIH arrhythmia database are used for test set, and there is no intersection between the training data set and test data set. The experimental data statistics can be seen from Table 1. The common heartbeat category example is shown in Figure 10.

### 5.2. Evaluation Measurement

As shown in formulas (14)–(17), TP, FP, TN, and FN need to be calculated in this paper to get the result of heartbeat classification. Among them, TP_*N*_ represents N category true-positive heartbeat, FP_*N*_ represents N category false-positive heartbeat, TN_*N*_ represents N category true-negative heartbeat, and FN_*N*_ represents *N* category false-negative heartbeat. The classification results of other categories of heartbeat are calculated in the same way [39].  Table 2 shows the confusion matrix of classification results, where, N, S, V, F, Q represent the real type of heartbeat, and *n*, *s*, *v*, *f*, *q* represent the predicted result.

(14) $$\begin{array}{c} {\text{TP}}_{N}=N_{n}, \end{array}$$

(15) $$\begin{array}{c} {\text{FP}}_{N}=N_{s}+N_{v}+N_{f}+N_{q}, \end{array}$$

(16) $$\begin{array}{c} {\text{TN}}_{N}=S_{s}+S_{v}+S_{f}+S_{q}+V_{s}+V_{v}+V_{f}+V_{q}+F_{s}+F_{v}+F_{f}+F_{q}+Q_{s}+Q_{v}+Q_{f}+Q_{q}, \end{array}$$

(17) $$\begin{array}{c} {\text{FN}}_{N}=S_{n}+V_{n}+F_{n}+Q_{n}. \end{array}$$

In this paper, sensitivity, specificity, positive predictivity, and accuracy are used to evaluate the performance of classifiers [39]. Sensitivity (Se) refers to the proportion of samples judged as positive cases in all positive cases. Specificity (Sp) refers to the proportion of samples judged as negative cases in all negative cases. The positive predictive value (*+p*) is also known as precision. Accuracy (Acc) is the ratio of correctly classified samples to total samples. The calculation formulas (18)–(21) for the above four evaluation indicators are as follows:

(18) $$\begin{array}{c} \text{Se}=\frac{\text{TP}}{\text{TP}+\text{FN}}, \end{array}$$

(19) $$\begin{array}{c} \text{Sp}=\frac{\text{TN}}{\text{TN}+\text{FP}}, \end{array}$$

(20) $$\begin{array}{c} +p=\frac{\text{TP}}{\text{TP}+\text{FP}}, \end{array}$$

(21) $$\begin{array}{c} \text{Acc}=\frac{\text{TP}+\text{TN}}{\text{TP}+\text{TN}+\text{FP}+\text{FN}}. \end{array}$$

### 5.3. Test Results of Different Feature Combinations

Feature selection is the most effective way to eliminate irrelevant dimensions. In order to compare the effects of different features on the classification of heartbeat, while ensuring the classification performance of the feature vector, considering the system complexity, this project conducted multiple tests using the set A, B, C, D, E with Adaboost + Random Forest models to select the best combination of features. In total, 16 tests are conducted. Among them, tests (1) –(5) compare the effect of single feature classification; tests (6)–(11) compare the classification effect of the pairwise combination of features; tests (12)–(15) compare the classification effect of three-feature combination; test (16) compares the classification effect of four-feature combination. The final result is that for Adaboost + RF, as the number of feature combinations increases, the accuracy is on the rise. Test (17) compares the performance difference between Adaboost + RF and other base classifiers under different feature combinations.

Test (1) conducted heartbeat classification using AdaBoost + Random Forest model with set A. The test is performed on 235 feature points in a single heartbeat. The results show that the average accuracy of classification is 98.59%.  Table 3 shows the classification results of AdaBoost + Random Forest model tested on the 235 single heartbeat morphological features. Test (2) classified heartbeat based on set B. The results show that the average accuracy of heartbeat classification is 98.84%.  Table 4 shows the classification results of the test on the 470 single heartbeat morphological features. Compared with test (1), the results showed that two leads morphology feature is more sufficient than that of the single lead. Test (3) classified heartbeat based on set C. The results show that the average accuracy of classification is 94.37%. But, the sensitivity and positive predictive value of F category are lower.  Table 5 shows the classification results of the test on the interval features. The disadvantage of test (3) is that the classification of heartbeat based on interval information alone is not obvious. Test (4) classified heartbeat based on set D. The results show that the sensitivity and positive predictive values of S, V, F, and Q heartbeat are lower, and the average classification accuracy is only 79.92%.  Table 6 shows the classification results of the test on the QRS area. The disadvantage of test (4) is that it has poor discrimination only according to QRS area. In test (5), the heartbeat is classified based on set E. The test results show that the sensitivity of S category and F category is low, and the average classification accuracy is 94.68%.  Table 7 shows the classification results of the test on the wavelet coefficient. Only using wavelet coefficients cannot describe the heartbeat signal completely, and it is difficult to distinguish the heartbeat with shape close to each other.

Test (6) classified heartbeat based on set B, C. The test results show that the average classification accuracy is 98.97%.  Table 8 shows the classification results of the test on the 470 single heartbeat morphological features and interval feature. Compared with test (2) and test (3), the sensitivity of S category and F category recognition is improved. In test (7), the heartbeat is classified based on set B, D. The test results show that the average classification accuracy is 98.83%.  Table 9 shows the classification results of the test on the 470 single heartbeat morphological features and QRS area. Compared with test (6), it can be seen that the interval features are superior to QRS area information in distinguishing S and F heartbeat types. Test (8) classified heartbeat based on set B, E. The results show that the average classification accuracy is 98.15%. But, the sensitivity of S category and F category is low. They are only 58.49% and 67.09%, respectively.  Table 10 shows the classification results of the test on the 470 single heartbeat morphological features and wavelet coefficient. Compared with test (6) and test (7), the deficiency of this feature combination is the lack of interval features, which is an important basis for judging S category and F category of heartbeat. In test (9), the heartbeat is classified based on set C, D. The results show that the average accuracy of classification is 96.59%, but the sensitivity of F category heartbeat is only 39.24%.  Table 11 shows the classification results of the test on the interval feature and QRS area. Compared with test (7), it can be seen that it is better to use the 470 single heartbeat morphological features to distinguish F category heartbeat. Test (10) classified heartbeat based on set C, E. The test results show that the average classification accuracy is 98.51%.  Table 12 shows the classification results of the test on the wavelet coefficient and interval feature. However, this kind of feature combination cannot effectively distinguish morphologically similar categories of heartbeat, such as N, S category, or V, F category. In test (11), the heartbeat is classified based on set D, E. The results show that the average accuracy of heartbeat classification is 98.24%.  Table 13 shows the classification results of the test on the QRS area and wavelet coefficient. Similar to the test (10), this feature combination also cannot effectively distinguish morphologically similar categories of heartbeat.

Test (12) classified heartbeat based on set B, C, D. The test (12) results show that the average classification accuracy is 99.09%.  Table 14 shows the classification results of the test on the interval feature, QRS area, and the 470 single heartbeat morphological features. Compared with test (9), the 470 single heartbeat morphological features can effectively improve the overall recognition rate of heartbeat classification. Test (13), heartbeat is classified based on set B, C, E. The average accuracy of this experiment is 99.00%.  Table 15 shows the classification results of the test on the 470 single heartbeat morphological features, interval feature, and wavelet coefficient. Compared with test (14), the interval features are slightly better than QRS area in overall classification performance. In test (14), the heartbeat is classified based on set B, D, E. The test (14) results show that the sensitivity of S category and F category heartbeat is not high, and the average accuracy of classification is 98.92%.  Table 16 shows the classification results of the test on the 470 single heartbeat morphological features, QRS area, and wavelet coefficient. Compared with test (16), the disadvantage of this experiment is the lack of interval feature, which is an important basis for improving the judgment of heartbeat category. In test (15), the heartbeat is classified based on set C, D, E. The test results show that the average accuracy of classification is 98.44%.  Table 17 shows the classification results of the test on the interval feature, QRS area, and wavelet coefficient. Compared with test (16), it is necessary to use the 470 single heartbeat morphological features to distinguish heartbeat categories. In test (16), heartbeat is classified based on set B, C, D, E. The test results show that the average classification accuracy is 99.11%.  Table 18 shows the classification results of the test on the 470 single heartbeat morphological features, interval features, QRS area, and wavelet coefficient. All the above experiments show that the optimal feature combination is set B, C, D, E.  Figure 11 presents the classification results and performance of the optimal feature combination with AdaBoost + Random Forest model.

As the tree (n_estimators) in the random forest of the base classifier is random, different classification results will be produced when different number of parameters are set. Generally, the number of parameters is too small to fit; and the number of parameters is too large to improve the model significantly. Therefore, the parameter selection is very important.  Table 19 is the classification result using different number of parameters of the optimal feature combination. It can be seen from Table 19 that the performance of the classifier is the best when n_estimators are equal to 70.

The purpose of this experiment is to compare the classification performance of multiple classifiers and find that the random forest algorithm has a better recognition effect on the small sample types in the unbalanced experimental data in this article, so the random forest model is used as the basic classifier for AdaBoost ensemble learning. In test (17), the accuracy is used as the evaluation indicator to compare Gaussian Naive Bayes (GNB), Linear Discriminant Analysis (LDA), Decision Tree (DT), Random Forest (RF), Gradient Lifting Iterative Decision Tree (GBDT), Support Vector Machine (SVM), Logistic Regression (LR), and AdaBoost + Random Forest (AdaBoost + RF) model on different feature sets.  Table 20 presents the classification performance of different classifiers. It can be seen from among them that the LDA model also achieves the best result of 94.38% in set B, C, D, E. DT, RF, SVM, and LR models are based on set B, C, D to achieve the best classification effect. The accuracy is 97.85%, 99.08%, 99.04% and 95.87%, respectively. GNB model achieved the best classification result of 85.39% based on set D, and GDBT model achieved the best classification effect based on set B, C,E. The best classification result is based on AdaBoost + Random Forest model with set B, C, D, E. The average accuracy of the classification is 99.11%. In this paper, after comparing the classification performance of these classifiers under each feature combination, the Random Forest with the best performance is selected as the base classifier for ensemble learning. Tests (1)–(16) are the detailed results of the classification of AdaBoost + Random Forest.

### 5.4. Comparative Results with Other Implemented Classification Methods

The system developed in this paper performs better on classification indicators [43, 51–54].  Table 21 presents comparison with previous studies. Compared with references [21, 55–58], the sensitivity and positive predictive value of N, S, and V heartbeats have been greatly improved. Compared with other methods, the accuracy of heartbeat classification is improved. The experimental results show that the method has the advantages of distinguishing N (nonectopic beats), V (ventricular ectopic beats), and Q (unknown beats). AdaBoost + Random Forest model is used to classify arrhythmia, and an accurate and objective heartbeat analysis system is established.

### 5.5. Clinical Data Test

In order to verify the actual effect, real data were collected for testing. The disease tag is the result given by the doctor. The format is float, 32 bit binary format, the sampling rate is 1000, and each data have 12 leads.  Figure 12 is the presented results of the ECG classification. Therefore, this system has evident clinical significance and practical value in the diagnosis of arrhythmia.

## 6. Conclusion

A novel, effective system of arrhythmia classification based on multi-feature fusion with optimal feature selection using AdaBoost + Random Forest model is presented in this paper. Based on this system, doctors can check the similarity and difference in features through machine learning model. The classification system of arrhythmia proposed in this paper has high recognition rate and is of great significance in clinical application. Although cardiac classification has made significant progress in the diagnosis of cardiovascular diseases, the sensitivity of this method of S and F category heartbeat needs to be improved. In order to achieve better classification effect, the future research will focus on improving the recognition performance of S and F category heartbeat.

Highlights of this paper are as follows:

1. This system accomplished automation from ECG signal collection, intelligent analysis to result presentation, thereby effectively improving the efficiency of doctor's diagnosis.
2. In the case of unbalanced ECG data set, a novel AdaBoost + Random Forest approach is proposed for the heartbeat classification system.
3. The framework is used to learn the potential correlation between an individual heartbeat internal data and the relationship of the different individual heartbeats.
4. Among a total 8 of classifiers examined, the AdaBoost + Random Forest is capable of achieving the best on the obtained optimal feature set.

## Figures and Tables

**Figure 1:** The overall architecture of the system.

**Figure 2:** The logic design of the system.

**Figure 3:** The ECG system function diagram.

**Figure 4:** The framework of heartbeat classification algorithm.

**Figure 5:** Example of two leads (II, V1) in an MIT-BIH arrhythmia database record 210 (10 sec).

**Figure 6:** Interval diagram of normal heartbeat.

**Figure 7:** The decomposition process of the 12-level wavelet packet (a).

**Figure 8:** The decomposition process of the 12-level wavelet packet (b).

**Figure 9:** The process of generating the final classifier.

**Figure 10:** Common heartbeat category example.

**Figure 11:** Confusion matrix of AdaBoost + Random Forest classification results tested on set B, C, D, E.

**Figure 12:** The result of clinical application of the algorithm.

**Algorithm 1:** AdaBoost ensemble algorithm steps.

**Table 1:** Experimental data statistics.

Category	Training set	Test set	Total
N	81,560	9,035	90,595
S	2,528	253	2,781
V	6,450	785	7,235
F	723	79	802
Q	7,248	793	8,041

**Table 2:** The confusion matrix of classification results.

	n	s	v	f	q

N	*N*_*n*_	*N*_*s*_	*N*_*v*_	*N*_*f*_	*N*_*q*_
S	*S*_*n*_	*S*_*s*_	*S*_*v*_	*S*_*f*_	*S*_*q*_
V	*V*_*n*_	*V*_*s*_	*V*_*v*_	*V*_*f*_	*V*_*q*_
F	*F*_*n*_	*F*_*s*_	*F*_*v*_	*F*_*f*_	*F*_*q*_
Q	*Q*_*n*_	*Q*_*s*_	*Q*_*v*_	*Q*_*f*_	*Q*_*q*_

**Table 3:** Performance of AdaBoost + Random Forest model tested on set A.

Prediction results						Evaluation standard (%)							
	n	s	v	f	q	TP	TN	FP	FN	Se	Sp	+p	Acc
N	9,030	1	4	0	0	9,030	1,776	134	5	99.94	92.98	98.53	98.73
S	51	199	1	0	2	199	10,691	1	54	78.65	99.99	99.50	99.49
V	45	0	739	1	0	739	10,144	16	46	94.14	99.84	97.88	99.43
F	19	0	10	50	0	50	10,865	1	29	63.29	99.99	98.03	99.74
Q	19	0	1	0	773	773	10,150	2	20	97.48	99.98	99.74	99.79

**Table 4:** Performance of AdaBoost + Random Forest model tested on set B.

Result						Evaluation criteria (%)							
	n	s	V	f	q	TP	TN	FP	FN	Se	Sp	+p	Acc
N	9,035	0	0	0	0	9,035	1,793	117	0	1.0	93.87	98.72	98.93
S	58	195	0	0	0	195	10,692	0	58	77.07	1.0	1.0	99.47
V	36	0	749	0	0	749	10,150	10	36	95.41	99.90	98.68	99.57
F	13	0	10	56	0	56	10,866	0	23	70.88	1.0	1.0	99.79
Q	10	0	0	0	783	783	10,152	0	10	98.74	1.0	1.0	99.91

**Table 5:** Performance of AdaBoost + Random Forest model tested on set C.

Result						Evaluation criteria (%)							
	n	s	v	F	q	TP	TN	FP	FN	Se	Sp	+p	Acc
N	8,926	21	36	11	41	8,926	1,458	452	109	98.79	76.33	95.18	94.87
S	88	156	6	0	3	156	10,666	26	97	61.66	99.75	85.71	98.87
V	180	5	578	2	20	578	10,100	60	207	73.63	99.41	90.59	97.56
F	52	0	8	18	1	18	10,853	13	61	22.78	99.88	58.06	99.32
Q	132	0	10	0	651	651	10,087	65	142	82.09	99.36	90.92	98.10

**Table 6:** Performance of AdaBoost + Random Forest model tested on set D.

Result						Evaluation criteria (%)							
	n	s	v	f	q	TP	TN	FP	FN	Se	Sp	+p	Acc
N	8,235	173	226	33	368	8,235	764	1,146	800	91.15	40.00	87.78	82.22
S	202	30	9	0	12	30	10,505	187	223	11.86	98.25	13.82	96.25
V	339	6	341	13	86	341	9,817	343	444	43.44	96.62	49.85	92.81
F	62	0	11	2	4	2	10,814	52	77	2.53	99.52	3.70	98.82
Q	543	8	97	6	139	139	9,682	470	654	17.53	95.37	22.82	89.73

**Table 7:** Performance of AdaBoost + Random Forest model tested on set E.

Result						Evaluation criteria (%)							
	n	s	V	f	q	TP	TN	FP	FN	Se	Sp	+p	Acc
N	9,034	0	1	0	0	9,034	1,337	573	1	99.98	70.00	94.43	94.76
S	206	47	0	0	0	47	10,692	0	206	18.85	1.0	1.0	98.11
V	217	0	568	0	0	568	10,151	9	217	72.36	99.91	98.44	97.94
F	47	0	8	24	0	24	10,866	0	55	30.38	1.0	1.0	99.50
Q	103	0	0	0	690	690	10,152	0	103	87.01	1.0	1.0	99.05

**Table 8:** Performance of AdaBoost + Random Forest model tested on set B, C.

Result						Evaluation criteria (%)							
	n	s	v	f	q	TP	TN	FP	FN	Se	Sp	+p	Acc
N	9,035	0	0	0	0	9,035	1,809	101	0	1.0	94.71	98.89	99.08
S	49	203	1	0	0	203	10,692	0	50	80.24	1.0	1.0	99.54
V	29	0	754	2	1	754	10,150	10	31	96.05	99.90	98.70	99.63
F	13	0	9	57	0	57	10,864	2	22	72.15	99.98	96.61	99.78
Q	10	0	0	0	783	783	10,152	0	10	98.74	1.0	1.0	99.91

**Table 9:** Performance of AdaBoost + Random Forest model tested on set B, D.

Result						Evaluation criteria (%)							
	n	s	v	f	q	TP	TN	FP	FN	Se	Sp	+p	Acc
N	9,034	1	0	0	0	9,034	1,796	114	1	99.99	94.03	98.75	98.95
S	59	192	2	0	0	192	10,691	1	61	75.89	99.99	99.48	99.43
V	30	0	753	2	0	753	10,149	11	32	95.92	99.89	98.56	99.61
F	15	0	9	55	0	55	10,864	2	24	69.62	99.98	96.49	99.76
Q	10	0	0	0	783	783	10,152	0	10	98.73	1.0	1.0	99.91

**Table 10:** Performance of AdaBoost + Random Forest model tested on set B, E.

Result						Evaluation criteria (%)							
	n	s	v	f	q	TP	TN	FP	FN	Se	Sp	+p	Acc
N	9,035	0	0	0	0	9,035	1,718	192	0	1.0	89.95	97.92	98.25
S	105	148	0	0	0	148	10,692	0	105	58.49	1.0	1.0	99.05
V	51	0	733	1	0	733	10,151	9	52	93.37	99.91	98.78	99.45
F	17	0	9	53	0	53	10,865	1	26	67.09	99.99	98.15	99.75
Q	19	0	0	0	774	774	10,152	0	19	97.60	1.0	1.0	99.83

**Table 11:** Performance of AdaBoost + Random Forest model tested on set C, D.

Result						Evaluation criteria (%)							
	n	s	v	f	q	TP	TN	FP	FN	Se	Sp	+p	Acc
N	8,985	5	26	4	15	8,985	1,617	293	50	99.44	84.66	96.84	96.86
S	70	168	15	0	0	168	10,687	5	85	66.40	99.95	97.11	99.18
V	98	0	683	0	4	683	10,108	52	102	87.01	99.48	92.93	98.59
F	39	0	9	31	0	31	10,862	4	48	39.24	99.96	88.57	99.52
Q	86	0	2	0	705	705	10,133	19	88	88.90	99.81	97.37	99.02

**Table 12:** Performance of AdaBoost + Random Forest model tested on set C, E.

Result						Evaluation criteria (%)							
	n	s	v	f	q	TP	TN	FP	FN	Se	Sp	+p	Acc
N	9,025	0	10	0	0	9,025	1,779	131	10	99.89	93.14	98.57	98.71
S	57	192	4	0	0	192	10,692	0	61	75.89	1.0	1.0	99.44
V	31	0	752	2	0	752	10,130	30	33	95.79	99.70	96.16	99.42
F	15	0	15	49	0	49	10,864	2	30	62.02	99.98	96.08	99.71
Q	28	0	1	0	764	764	10,152	0	29	96.34	1.0	1.0	99.74

**Table 13:** Performance of AdaBoost + Random Forest model tested on set D, E.

Result						Evaluation criteria (%)							
	n	s	v	f	q	TP	TN	FP	FN	Se	Sp	+p	Acc
N	9,025	0	10	0	0	9,025	1,743	167	10	99.89	91.25	98.18	98.38
S	78	174	1	0	0	174	10,692	0	79	68.77	1.0	1.0	99.27
V	46	0	738	1	0	738	10,135	25	47	94.01	99.75	96.72	99.34
F	16	0	14	49	0	49	10,865	1	30	62.03	99.99	98.00	99.72
Q	27	0	0	0	766	766	10,152	0	27	96.59	1.0	1.0	99.75

**Table 14:** Performance of AdaBoost + Random Forest model tested on set B, C, D.

Result						Evaluation criteria (%)							
	n	s	v	f	q	TP	TN	FP	FN	Se	Sp	+p	Acc
N	9,030	2	3	0	0	9,030	1,828	82	5	99.94	95.71	99.10	99.20
S	40	211	2	0	0	211	10,690	2	42	83.40	99.98	99.06	99.59
V	23	0	761	1	0	761	10,145	15	24	96.94	99.85	98.07	99.64
F	11	0	10	58	0	58	10,865	1	21	73.42	99.99	98.31	99.80
Q	8	0	0	0	785	785	10,152	0	8	98.99	1.0	1.0	99.93

**Table 15:** Performance of AdaBoost + Random Forest model tested on set B, C, E.

Result						Evaluation criteria (%)							
	n	s	v	f	q	TP	TN	FP	FN	Se	Sp	+p	Acc
N	9,028	3	4	0	0	9,028	1,820	90	7	99.92	95.29	99.01	99.11
S	44	207	2	0	0	207	10,689	3	46	81.82	99.97	98.57	99.55
V	25	0	760	0	0	760	10,144	16	25	96.82	99.84	97.94	99.63
F	13	0	10	55	1	55	10,866	0	24	69.62	1.0	1.0	99.78
Q	8	0	0	0	785	785	10,151	1	8	98.99	99.99	99.87	99.92

**Table 16:** Performance of AdaBoost + Random Forest model tested on set B, D, E.

Result						Evaluation criteria (%)							
	n	s	v	f	q	TP	TN	FP	FN	Se	Sp	+p	Acc
N	9,028	2	5	0	0	9,028	1,811	99	7	99.92	94.82	98.92	99.03
S	56	197	0	0	0	197	10,690	2	56	77.87	99.98	98.99	99.47
V	21	0	764	0	0	764	10,143	17	21	97.32	99.83	97.82	99.65
F	12	0	12	55	0	55	10,866	0	24	69.62	1.0	1.0	99.78
Q	10	0	0	0	783	783	10,152	0	10	98.74	1.0	1.0	99.91

**Table 17:** Performance of AdaBoost + Random Forest model tested on set C, D, E.

Result						Evaluation criteria (%)							
	n	s	v	f	q	TP	TN	FP	FN	Se	Sp	+p	Acc
N	9,025	0	9	0	1	9,025	1,763	147	10	99.89	92.30	98.89	98.56
S	64	189	0	0	0	189	10,692	0	64	74.70	1.0	1.0	99.42
V	36	0	748	1	0	748	10,138	22	37	95.28	99.78	97.14	99.46
F	18	0	11	50	0	50	10,865	1	29	63.29	99.99	98.04	99.73
Q	29	0	2	0	762	762	10,151	1	31	96.09	99.99	99.87	99.71

**Table 18:** Performance of AdaBoost + Random Forest model tested on set B, C, D, E.

Result						Evaluation criteria (%)							
	n	s	v	f	q	TP	TN	FP	FN	Se	Sp	+p	Acc
N	9,031	1	3	0	0	9,031	1,837	79	4	99.95	95.86	99.13	99.24
S	43	209	1	0	0	209	10,691	1	44	82.61	99.99	99.52	99.58
V	20	0	765	0	0	765	10,144	16	20	97.45	99.84	97.95	99.67
F	10	0	12	56	1	56	10,866	0	23	70.88	1.0	1.0	99.79
Q	6	0	0	0	787	787	10,151	1	6	99.24	99.99	99.87	99.94

**Table 19:** Classification results of different (n_estimators) numbers.

Parameter (n_estimators)	20	30	40	50	60	70	80	90
Accuracy (%)	98.34	98.25	98.28	98.29	99.07	**99.11**	99.10	99.08

**Table 20:** Accuracy of different classifiers performed with multiple-feature combinations.

Feature set					Classifiers							
A	B	C	D	E	GNB	LDA	LR	SVM	DT	GBDT	RF	**Adaboost** + **RF**
*∗*					49.05	90.05	91.81	98.68	97.09	97.65	98.64	98.59
	*∗*				55.86	92.79	93.94	98.96	97.73	98.37	98.91	98.84
		*∗*			82.06	82.69	82.85	91.89	91.51	91.83	94.45	94.37
			*∗*		**85.39**	82.55	82.55	85.42	79.62	85.55	79.15	79.92
				*∗*	83.04	90.19	91.86	96.88	96.49	97.65	98.17	94.68
	*∗*	*∗*			56.38	93.31	94.47	99.00	97.73	98.53	98.91	98.97
	*∗*		*∗*		69.63	92.77	93.92	98.96	97.78	98.39	99.02	98.83
	*∗*			*∗*	69.14	92.76	93.92	98.51	97.41	98.53	98.92	98.15
		*∗*	*∗*		85.23	83.99	85.05	95.08	94.23	94.66	96.88	96.59
		*∗*		*∗*	84.09	92.19	93.60	97.25	96.98	98.14	98.43	98.51
			*∗*	*∗*	83.03	90.24	91.88	96.91	96.65	97.60	98.16	98.24
	*∗*	*∗*	*∗*		56.63	94.16	**95.87**	**99.04**	**97.85**	98.66	**99.08**	99.09
	*∗*	*∗*		*∗*	69.63	94.16	95.81	98.66	97.78	**98.70**	99.04	98.99
	*∗*		*∗*	*∗*	69.09	92.95	94.04	98.51	97.24	98.45	98.85	98.92
		*∗*	*∗*	*∗*	84.09	92.25	93.62	97.28	97.02	98.15	98.46	98.44
	*∗*	*∗*	*∗*	*∗*	69.59	**94.38**	95.82	98.66	97.73	98.64	99.00	**99.11**

**Table 21:** Comparison results with other implemented classification methods.

Reference	Features	Classifier	Performance
Zhang et al. [21]	ECG Morphology RR interval	SVM	Acc = 86.66%
			*Se*_*n*_ = 88.94%; *+P*_*n*_ = 98.98%
			*Se*_*s*_ = 79.06%; *+P*_*s*_ = 35.98%
			*Se*_*v*_ = 85.48%; +*P*_*v*_ = 92.75%
			*Se*_*f*_ = 93.81%; *+P*_*f*_ = 13.73%

Ghorbani Afkhami et al. [54]	HOS RR interval	DT	Acc = 99.70%
			*Se*_*n*_ = 97.37%; *+P*_*n*_ = 98.40%
			*Se*_*s*_ = 86.50%; *+P*_*s*_ = 90.90%
			*Se*_*v*_ = 95.99%; +*P*_*v*_ = 77.63%
			*Se*_*f*_ = 11.86%; *+P*_*f*_ = 24.21%

Yang et al. [53]	PCAnet	LinearSVM	Acc = 97.77%
			*+P*_*n*_ = 98.05%
			*+P*_*s*_ = 92.80%
			+*P*_*v*_ = 94.59%
			*+P*_*f*_ = 91.75%
			*+P*_*q*_ = 99.50%

Wang et al. [43]	Medical features	RF	Acc = 99.08%
	Statistical features		
	Morphological features		

Ji et al. [56]	ECG morphology	Faster R-CNN	Acc = 99.21%
			Se = 98.06%; Sp = 99.45%

Sharma et al. [57]	Morphological features	KNN	Acc = 98.10%
	Wavelet transform		*Se*_*n*_ = 99.59%; *Sp*_*n*_ = 91.92%; *+P*_*n*_ = 98.34%
			*Se*_*s*_ = 73.64%; *Sp*_*s*_ = 99.84%; *+P*_*s*_ = 92.09%
			*Se*_*v*_ = 92.11%; *Sp*_*v*_ = 99.75%; +*P*_*v*_ = 96.37%
			*Se*_*f*_ = 64.46%; *Sp*_*f*_ = 99.94% *+P*_*f*_ = 88.38%

Li et al. [58]	RR intervals Morphological features	CraftNet	Acc = 89.25%
			*Se*_*n*_ = 88.16%; *Sp*_*n*_ = 94.34%
			*Se*_*s*_ = 85.37%; *Sp*_*s*_ = 94.85%
			*Se*_*v*_ = 94.53%; *Sp*_*v*_ = 99.70%
			*Se*_*f*_ = 88.92%; *Sp*_*f*_ = 94.28%

Proposed	ECG morphology	AdaBoost + RF	Acc = 99.11%
	Intervals		*Se*_*n*_ = 99.95%; *Sp*_*n*_ = 95.86%; *+P*_*n*_ = 99.13%
	QRS area		*Se*_*s*_ = 82.61%; *Sp*_*s*_ = 99.99%; *+P*_*s*_ = 99.52%
	Wavelet coefficients		*Se*_*v*_ = 97.45%; *Sp*_*v*_ = 99.84%; +*P*_*v*_ = 97.95%
			*Se*_*f*_ = 70.88%; *Sp*_*f*_ = 100%; *+P*_*f*_ = 100%
			*Se*_*q*_ = 99.24%; *Sp*_*q*_ = 99.99%; *+P*_*q*_ = 99.87%

## Data Availability

(1) All data sets used to support the findings of this study are included within the paper. (2) All data sets used to support the findings of this study were supplied by the publicly available MIT-BIH database from the Massachusetts Institute of Technology. The URL to access this data is https://www.physionet.org/cgi-bin/atm/ATM. (3) The coding used to support the findings of this study have not been made available because the source code in this paper is part of a national project and is a trade secret; hence, the source code is not available.
